# Measuring Latency Variations in Evoked Potential Components Using a Simple Autocorrelation Technique

**DOI:** 10.1155/2021/8875445

**Published:** 2021-09-22

**Authors:** Jackie Campbell, Massimo Leandri

**Affiliations:** ^1^Faculty of Health, Education and Society, University of Northampton, Northampton NN1 5PH, UK; ^2^Dipartimento di Neuroscienze (DINOGMI), Università Degli Studi di Genova, Genova I-16132, Italy

## Abstract

Interpretation of averaged evoked potentials is difficult when the time relationship between stimulus and response is not constant. Later components are more prone to latency jitter, making them insufficiently reliable for routine clinical use even though they could contribute to greater understanding of the functioning of polysynaptic components of the afferent nervous system. This study is aimed at providing a simple but effective method of identifying and quantifying latency jitter in averaged evoked potentials. Autocorrelation techniques were applied within defined time windows on simulated jittered signals embedded within the noise component of recorded evoked potentials and on real examples of somatosensory evoked potentials. We demonstrated that the technique accurately identifies the distribution and maximum levels of jitter of the simulated components and clearly identifies the jitter properties of real evoked potential recording components. This method is designed to complement the conventional analytical methods used in neurophysiological practice to provide valuable additional information about the distribution of latency jitter within an averaged evoked potential. It will be useful for the assessment of the reliability of averaged components and will aid the interpretation of longer-latency, polysynaptic components such as those found in nociceptive evoked potentials.

## 1. Introduction

Clinical neurophysiology uses potentials recorded from the human scalp, evoked by peripheral stimulation, to investigate the integrity of the neural pathways of various sensory modalities [1]. The conventional form of analysis is a simple average, where the stimulus is repeated multiple times and the recording process is triggered by the stimulus onset. Each successive recording is added to the previous ones, with appropriate adjustment of amplitude, to form a running average. This process assumes that the signal components of interest are time-locked to the stimulus onset, whereas the background noise is assumed to be random with respect to the stimulus. Consequently, as increasing numbers of recordings are added to the average, the noise elements reduce whilst the signal components retain their original amplitude and are seen to “grow” out of the background noise. In theory, an average of an infinite number of recordings would have zero noise, and the signal would be revealed with its true amplitude [2].

However, the underlying neurophysiology of the production of the evoked potential (EP) is not compatible with the assumptions of averaging. In particular, there is evidence that evoked potential components vary in both amplitude and latency on repeated recordings, with later components displaying greater latency variations (“jitter”) [3]. Signal components which occur at the same point in time relative to the stimulus onset but have different amplitudes produce averaged components of identical shape and latency but varying amplitudes. When different signal components overlap in time, they will produce shape changes in the composite signal, but the latencies of the individual components will not change. However, varying latencies within a single signal component can also produce shape and amplitude distortions, but the apparent latency as measured on the averaged signal will not be a true measure of the original signals.

Early components of scalp-recorded evoked potentials represent activity from fast neural pathways, which only have a few synapses and therefore have the least latency variation. This makes them sufficiently consistent and reliable for clinical use [4]. However, the later components are susceptible to much greater variability because of the larger number of synapses and involvement with other aspects of brain responses, such as attention. In addition, some modalities of stimulation, such as for visual and auditory evoked potentials, do not achieve the same synchronous volley as that produced by electrical stimulation of fast sensory afferent fibres, which also results in variability in the latency of the recorded components [5]. Nociceptive evoked potentials are a comparatively new addition to the potential tools for examining the nervous system and are mediated by slow peripheral fibres in addition to undergoing numerous synapses [6]. This and the limited number of repetitions of the stimulus that are possible have resulted in their use in only very limited clinical settings.

A previous study by the authors [7] describes a method of assessing the reliability of an averaged evoked potential component, using the median correlation coefficient of pairs of repeated signals within specified time windows (median *r*). This technique quantifies the similarity in shape of the evoked potential produced by each external stimulus, within specified time windows. Amplitude variation of discrete components alone does not affect the median *r* value. An averaged component with a high value of median *r* indicates that the constituent single responses are occurring at the same latency and have the same shape. Averaged components with low median *r* values could indicate either interference from other overlapping components unrelated to the stimulus or that the single responses have variation in latency. This study extends the utility of this approach by additionally identifying the distribution of the latency shift exhibited by any specified component. The proposed analysis technique could be performed in parallel with the acquisition of conventionally averaged responses and can give important additional information about the role of latency variability in components with low signal reliability. In addition, information about the nature of latency variation may be relevant for both clinical and research contexts [8].

Other methods have been used to take account of latency jitter of EP components: Achimowicz [9], for example, used phase domain pattern recognition techniques; Hu et al. [10] used wavelet filtering together with multiple linear regression; Limpiti et al. [11] used an expectation-maximisation algorithm; and Mayhew et al. [12] used multiple linear regression techniques. However, these were all focussed on extraction of single trial EP characteristics in the presence of varying trial-to-trial latency, amplitude, and/or morphology of the components. The importance of investigating the latency properties of EPs was recognised by Woody [13], who developed an iterative adaptive filter which used autocorrelations between the averaged response and each individual record to align the components on the time axis and calculate a new average. This process was repeated until there was no change between iterations. The method was refined by Thornton [14] using subaverages. A refinement of Woody's algorithm [13], incorporating the maximum likelihood technique, has also been used [15]. Ma et al. [8] recognised the clinical utility of latency jitter and used independent component analysis (ICA) of multichannel recordings to compare jitter in animal studies. None of these techniques are in common clinical use, however. This study takes a simple approach to the identification of the distribution of latency changes of a defined EP component to give information on the latency variability, which is easily interpreted and can be used alongside the conventional averaged response in clinical practice.

## 2. Materials and Methods

Somatosensory evoked potentials (SEPs) were recorded, with informed consent, from two neurologically normal subjects. These were used as genuine biological samples in the testing of the autocorrelation method. SEPs were obtained after surface stimulation of the median nerve at the right wrist, with 0.2 ms electric pulses delivered at the rate of 0.83 Hz and intensity set at the threshold for thumb twitch. Recordings were performed from C3′-Fz scalp derivation with surface electrodes, where C3′ is the usual upper limb SEP recording position, over the hand projection in the sensory homunculus [16]. The same electrodes were used to record equivalent time epochs of EEG spontaneous activity, without any stimulation (called SEP noise later in this paper). Amplification of ×100,000 was used with a bandpass of 0.1-2,000 Hz, using 2nd-order Butterworth analog filtering (LT amplifiers by Vertigo, Genova, Italy). Signals were then sent to an analog-to-digital converter (NI PCIe-6320, X Series Multifunction DAQ, 16 bit, 250 kHz sampling rate by National Instruments, Austin, Texas). Software was developed using LabView 2017® (National Instruments, Austin, Texas) to acquire 10,000 samples for a period of 1,000 ms after each stimulus, thus providing a high definition recording with a dwell time of 0.1 ms. Each response was stored on a hard disc for off-line averaging.

Simulated single evoked potential components were constructed using NI LabView 2017® [17], based on the generation of a sine wave with variable width and -90° phase shift at a given distance along the time axis. Jitter (uncertainty in peak latency) was simulated by applying a random shift along the time axis, within given maximum limits, every time the sinusoid was generated and summing the specified number of iterations. The total length of the simulated signal was 1,000 ms with a dwell time of 0.1 ms (data acquisition rate of 10 kHz) for compatibility with the parameters used in the SEP recordings described above. Amplitude and DC shift were constant within the simulation program, but adjustable between simulations.

Autocorrelation methods were used for identification of latency jitter. Autocorrelation is a method which can identify similar signals that are delayed in time with respect to each other [18]. For this study, a time window of interest was defined in the averaged evoked potential recording. Pairs of single response records were used to calculate the correlation coefficient between them. This was initially calculated with both records starting at the same time point. A constant time shift was then introduced by moving one record along the time axis relative to the other by a constant amount and recalculating the correlation coefficient. This was repeated so the correlation coefficient was first calculated for both records starting at the same time point, then with the second record delayed by a time shift *δt*, then by time shift 2*δt*, etc., until the time shift was equal to the time window length. This was repeated for all possible pairs of records. This is illustrated in Figure 1.

A virtual instrument was constructed in LabView 2017 which identified a specified time window within a set of *N* repeated EP records, either real or simulated. An autocorrelation was then performed on every pair of records (a total of _*N*_*C*_2_ = *N*!/(2!(*N* − 2)!), using the LabView function crosscorrelation.vi, and the time difference for the maximum correlation for all pairs of records was plotted as a histogram.

## 3. Results and Discussion

### 3.1. Effect of Latency Shifts (“Jitter”) on Averaged Evoked Potential Components

Conventional signal averaging ideally requires a stationary signal and random noise in relation to the stimulus onset [2]. The median cross-correlation coefficient of every possible pair of repeated signals (median *r*) within a defined time window has been used as a measure of the reliability of signal components where reliability is defined in terms of repeatability [7]. As change in amplitude alone does not alter the median *r*, this reliability is therefore expressed as components of similar shape occurring at the same latency. However, there is evidence that evoked potential components vary in both amplitude and latency, with later components displaying greater latency variations (“jitter”) [3]. This section, therefore, looks at the effect of varying amounts of jitter on the averaged components and their reliability (as measured by median *r*), using simulated signal components.

Figure 2 shows an example of a simulated EP component with a peak latency of 100 ms, width at its base of 40 ms, and random jitter with a maximum of ±20 ms.  Figure 2(a) illustrates the jitter production (5 repetitions).  Figure 2(b) shows a single, unjittered simulated component, together with the compound potential produced by conventional averaging of 30 identical components with a jitter of ±20 ms. It can be seen that the presence of jitter affects the amplitude, shape, and latency of the averaged component.

Figure 3 shows the effect of latency jitter on an averaged simulated component within SEP noise of similar amplitude. The median *r* values for every 10 ms window are shown in red and are a measure of the repeatability of the signals within those windows (see above). The median *r* values of successive 10 ms windows rapidly decrease with increasing latency variation. With no jitter (Figure 3(a)), the simulated SEP component at c. 100 ms shows as a large amplitude peak amongst the averaged SEP noise, even though the amplitudes of the signal and the noise were similar for each of the 30 individual records. The median *r* value is high (>0.8), indicating that this component is highly reliable. When a small amount of jitter (±5 ms) is added to the simulated component (Figure 3(b)), the amplitude of the signal peak is smaller and broadened and the median *r* has decreased (c. 0.5), which reflects the increased unreliability of this component. With ±10 ms jitter (Figure 5(c)), the averaged signal is still visible, although again smaller and broader, but the median *r* is now indistinguishable from 0, indicating an unreliable signal component. This is an accurate representation if reliability of the averaged component is defined as representing a component of similar shape at the same latency. However, in the absence of further information, it may be indistinguishable from a single, large artefact, which would also give a low median *r*. Additional methods are needed to correctly interpret components which may be subject to latency jitter (see the next section).

### 3.2. Identifying and Measuring Latency Jitter in Individual Components

An autocorrelation was performed to investigate latency jitter in specified components. A specified time window was defined to fit the component under investigation. The correlation coefficient between two records for this time window was calculated and repeated with one of the records successively time-shifted by a specified amount (by default, this was the dwell time of the recording). The time shift that produced the highest correlation coefficient was recorded, and this was repeated for every possible dissimilar pair of records. The results were displayed as a histogram of the time shifts that produced the maximum correlation for all possible pairs of records. The flow chart for this process is shown in Figure 1. This was first tested using simulated signals with known jitter and then on actual evoked potential recordings.

#### 3.2.1. Simulated Signals with Known Jitter

Figure 4 shows the results of performing an autocorrelation on 120 repetitions of the simulated signal shown in Figure 2, with a random, normally distributed jitter of up to ±10 ms applied to each signal. The time window was defined as 80-120 ms. The absolute time differences between the repetitions which gave the maximum correlation coefficient were plotted against the number of times this occurred between all possible dissimilar pairs of records (7,140 pairs of records when there are 120 repetitions). The shape of this histogram shows the distribution of the latency jitter. Absolute time differences were plotted on the *x*-axis, which is equivalent to reflecting the left (negative) portion of the distribution curve on to the positive portion. It can be clearly seen that the resulting measured latency shifts approximate to the positive portion of a normal distribution, reflecting the actual jitter distribution. The maximum time difference was 20 ms, which is equivalent to the ±10 ms jitter specified in the simulation.

Figure 5(a) uses the same small simulated signal (onset latency 90 ms, width 20 ms) with random jitter to a maximum of ±15 ms combined with recorded SEP noise of a similar amplitude. The resultant average of 30 records appears as a broadened peak with superimposed noise, and the median *r* (calculated for successive 50 ms time windows) goes from 0, where there is only noise, to approximately 0.05 for the width of the averaged signal, indicating poor reliability. However, the histogram from the autocorrelation (Figure 5(b)) clearly shows absolute time differences between similar peaks of up to 30 ms, which is equivalent to maximum jitter of ±15 ms. This knowledge of the presence of latency jitter (and its quantification) enables the low reliability of this component to be interpreted as representing a real signal component with latency jitter, rather than being due to a large artefact. A combination of cross-correlations (median *r*) and autocorrelation, therefore, gives an accurate representation of the underlying signal structure by enabling signal components with low reliability to be differentiated into those with large noise or artefacts (low median *r*, no autocorrelation) from those with repeatable, but latency shifted, components (low median, latency shifts identified).

#### 3.2.2. Using Recorded Somatosensory Potentials

Figure 6 shows the results of using both the cross-correlation (median *r*) and autocorrelation (peak difference detection) methods on a real somatosensory evoked potential (SEP) recording. The method of recording the SEP is detailed in Materials and Methods (section 2) Thirty repetitions were conventionally averaged and are shown in Figure 6(a). Three components of interest were identified lying in time windows 17-23 ms, 30-40 ms, and 45-80 ms (marked as A, B, and C in Figure 6(a)), and the median *r* values for these three time windows are superimposed on the averaged graph. The early component has a high median *r* value (c. 0.8), indicating high reliability in terms of both shape and latency. Figures 6(b)–6(d) look at windows A, B, and C, respectively, and present the distribution of the time interval that one record has to be time-shifted by to get maximum similarity with the shape of the other record in that pair. Each pair of records represents one count at that optimum time shift.  Figure 6(b) shows that the maximum time difference seen for component A was quite small at about 6 ms (which corresponds to a maximum latency jitter of ±3 ms). However, this natural jitter is not constrained to be normally distributed as was the case with the simulated signals, and most of the time, differences were less than 2 ms (±1 ms). Component B was associated with a median *r* value of c. 0.5, indicating worsening reliability, and this is confirmed by the results of the autocorrelation shown in Figure 6(c), which gives a slightly larger maximum latency jitter of 8 ms (±4 ms), with most being less than ±3 ms. The median *r* associated with the later component (C) was low, at 0.13. This is likely to be due to large latency variations, as verified in Figure 6(d), which shows a latency variation of up to 34 ms (±17 ms), with most being less than ±11 ms, for that component.

The time difference histograms shown in Figures 6(b)–6(d) give information about not only the maximum extent of the latency jitter but also the distribution of the time differences between repetitions of the signal. This could be a useful tool for investigating the nature of latency changes in research and clinical evoked potential applications.

## 4. Conclusions

This paper describes a simple way of adding latency variation (jitter) information to evoked potential components identified by conventional signal averaging. This is especially important for later components which are polysynaptic in origin and are therefore highly prone to variation in latency. The method described in this paper can quickly identify the distribution of latency variation and estimate the total jitter range.

The method used is intuitive and is designed to be used in conjunction with the conventional interpretation of the averaged evoked potential. It gives a clear, graphical indication of the distribution of the latency jitter of the recorded signal within any specified time window. This could be used, in conjunction with measures of component reliability [7], to identify and quantify those components whose low reliability is a result of latency shifts, rather than occasional, large artefacts. The jitter information could also be used to provide confidence intervals for conduction velocity measurements which rely on late evoked potential components after stimulation at different sites [19, 20]. Applying our method, a specified confidence interval of the latency jitter could easily be identified from analysis of the histogram of latency shifts, which can then be directly used to give the confidence interval of the conduction velocity related to that component. These can be compared statistically with normative ranges or between groups.

Latency jitter information would be particularly valuable when using nociceptive evoked potentials. The difficulty of reliably activating nociceptive pathways and the variability of amplitude and latency of the resultant evoked responses have limited the utility of this modality in clinical practice, although there is considerable evidence of their value [21–23]. However, recent advances in this field have included a new, reliable method of eliciting nociceptive evoked potentials [24–26], and this combination of improved recording technique and the analytical methods for quantification of reliability and latency jitter will enable these to be easily incorporated into future work to identify possible abnormalities of the afferent pathways or cortical processing.

## Figures and Tables

**Figure 1:** Flow chart of the autocorrelation method. *N* single response recordings of the evoked potential are used. For each possible, dissimilar pair of recordings *a* and *b* (of which there are _*N*_*C*_2_ = *N*!/(2!(*N* − 2)! combinations), an autocorrelation is performed within a specified time window (*t*_0_ to *t*_end_) by calculating the cross-correlation between the recordings (*r*_*i*_, where *i* identifies the unique pair of recordings). Recording *b* is then shifted along the time axis (relative to recording *a*) by a small amount *δt* (usually the dwell time of the recording), and the correlation is again calculated. This is repeated until recording *b* is shifted by the length of the time window. The time shift that produced the largest *r*_*i*_(*t*_*i*_) is then recorded, where *t*_*i*_ represents the latency shift between that pair of recordings. Another pair of recordings is then selected, and the process is repeated until all dissimilar pairs of recordings have been autocorrelated. The histogram of the *t*_*i*_s for all possible pairs shows the distribution of the latency jitter in the set of *N* responses.

**Figure 2:** Simulated EP components (peak latency 100 ms, width at base 40 ms). (a) shows 5 identical components with random jitter of ±20 ms. (b) shows a single, unjittered component (in red) together with the average (mean) of 30 identical components with random jitter of ±20 ms (blue). Amplitude is shown in arbitrary units.

**Figure 3:** Effect of latency jitter applied to a simulated single component with onset latency 90 ms and width 20 ms in recorded EP noise of similar amplitude. Averages of 30 recordings are shown together with the reliability measure (median *r*) for successive 10 ms windows with (a) no jitter, (b) random jitter of ±5 ms, and (c) random jitter of ±10 ms.

**Figure 4:** Histogram of the absolute time differences between pairs of records that produced the maximum correlation coefficient using 120 repetitions of a simulated signal of onset latency 90 ms and width 20 ms, with random jitter of a maximum of ±10 ms. Time window used was 80-120 ms.

**Figure 5:** (a) shows the average of 30 repetitions of the simulated signal (onset latency 90 ms, width 20 ms) with random jitter to a maximum of ±15 ms + SEP noise of similar amplitude, together with the reliability measure (median *r*) over 50 ms time windows. (b) shows the histogram of the peak time differences which gives maximum correlations for every dissimilar pair of 30 repetitions.

**Figure 6:** (a) An averaged somatosensory evoked potential (SEP) (average of 30 repetitions) recorded from the scalp (C_3_′-F_z_) after stimulation of the right median nerve at the wrist. Recorded from a neurologically normal female. Median *r* values (horizontal lines, right axis) are shown for three time windows which include identified signal components: A (17-23 ms), B (30-40 ms), and C (45-80 ms). (b), (c), and (d) are the autocorrelation histograms for the time windows for A, B, and C, respectively.

## Data Availability

All data used to support the findings of this study have been deposited in the University of Northampton PURE repository (doi:10.24339/432a276a-b10f-4adc-821a-b3a59fafb1a8).
